The article "Distributed Function Mining for Gene Expression Programming Based on Fast Reduction" was published in 2016. Journal: PLoS One.

# Distributed Function Mining for Gene Expression Programming Based on Fast Reduction

**DOI:** 10.1371/journal.pone.0146698

**Published:** 2016-01-11

**Authors:** Song Deng, Dong Yue, Le-chan Yang, Xiong Fu, Ya-zhou Feng

**Affiliations:** 1 Institute of Advanced Technology, Nanjing University Post & Telecommunication, Nanjing, 210023, China; 2 International Institute for Earth System Science, Nanjing University, Nanjing, 210093, China; 3 School of Computer, Nanjing University Post & Telecommunication, Nanjing, 210023, China; Cedars-Sinai Medical Center, UNITED STATES

## Abstract

For high-dimensional and massive data sets, traditional centralized gene expression programming (GEP) or improved algorithms lead to increased run-time and decreased prediction accuracy. To solve this problem, this paper proposes a new improved algorithm called distributed function mining for gene expression programming based on fast reduction (DFMGEP-FR). In DFMGEP-FR, fast attribution reduction in binary search algorithms (FAR-BSA) is proposed to quickly find the optimal attribution set, and the function consistency replacement algorithm is given to solve integration of the local function model. Thorough comparative experiments for DFMGEP-FR, centralized GEP and the parallel gene expression programming algorithm based on simulated annealing (parallel GEPSA) are included in this paper. For the waveform, mushroom, connect-4 and musk datasets, the comparative results show that the average time-consumption of DFMGEP-FR drops by 89.09%%, 88.85%, 85.79% and 93.06%, respectively, in contrast to centralized GEP and by 12.5%, 8.42%, 9.62% and 13.75%, respectively, compared with parallel GEPSA. Six well-studied UCI test data sets demonstrate the efficiency and capability of our proposed DFMGEP-FR algorithm for distributed function mining.

## Introduction

In practical applications, a function model that is mined from data sets helps to reveal the inherent nature of the data sets. Generally, traditional regression methods have assumed that the function type was known, and then, the least squares method or improved methods for parameter estimation were used to determine the functional model [1]. These traditional regression methods depended on a priori knowledge and many subjective factors. Moreover, these methods have high time complexity and low computational efficiency for complex and high-dimensional data sets. To solve these problems, Li et al. and Koza et al. used genetic programming (GP) for a mathematical model and obtained good experimental results [2,3]. At the same time, GP also avoided the defect in traditional statistical methods of selecting the function model in advance. However, the efficiency of the function model that was mined by GP was low. Thus, a new algorithm, which was called gene expression programming (GEP), was proposed [4]. Compared with GP, the efficiency of complex function mining based on GEP was increased by 4–6 times.

Currently, research on GEP is focused on the basic theory of the algorithms, symbolic regression, function mining, prediction and security assessment, among other topics.

**(1) Algorithm theory.** In algorithm theory, fitness distance correlation could only minimally predict the evolution difficulty of gene expression programming [5]. To solve this problem, Zheng et al. posed gene expression programming evolution difficulty prediction based on the posture model [5]. Zhu et al. present naive gene expression programming (NGEP) based on genetic neutrality, which was combined with the neutral theory of molecular evolution [6]. Extensive experiments showed that NGEP is more efficient than traditional GEP in the case of similar gene redundancy; in particular, the success rate of NGEP does not change drastically with the growth of genetic neutrality.

**(2) Symbolic regression and function mining.** In symbolic regression and function mining, Peng et al. proposed an improved GEP algorithm called S_GEP, which is especially suitable for addressing symbolic regression problems [7]. Experiments showed the powerful potential of S_GEP to address complex nonlinear symbolic regression problems. A new Prufer code optimization algorithm for multi-layer logistic networks based on gene expression programming was combined with the characteristics of the GEP multi-gene structure [8]. Experiments showed that the algorithm could obtain more convergence accuracy compared with traditional evolution algorithms. In view of the insufficiency of the existing forecasting model in highway construction cost forecasting, the highway construction cost forecasting model was proposed based on the GEP according to the characteristics of highway construction cost forecasting [9]. Experiment results demonstrated that the forecasting precision and application value of the model was high. To understand the treatment of marginal soil well, function finding via gene expression programming for the strength and elastic properties of clay treated with bottom ash was proposed [10]. Experiments showed that the GEP-based formulas for unconfined compressive strength and elasticity moduli are significantly capable of predicting the measured values to a high degree of accuracy against the nonlinear behavior of soil. Zhao et al. treated image registration as a formula discovery problem and proposed two-stage gene expression programming and the improved cooperative particle swarm optimizer, which they used to identify the registration formula for a reference image and floating image [11].

**(3) Prediction.** In prediction, Seyyed et al. present a new gene expression programming algorithm for the prediction model of electricity demand [12]. Chen et al. applied parallel hyper-cubic gene expression programming to estimate the slump flow of high-performance concrete [13]. Experiments showed that for estimating HPC slump flow, the parallel hyper-cubic GEP is more accurate than the traditional GEP and other regression models. Huo et al. applied gene expression programming to short-term load forecasting on power systems and proposed model error cycling compensation [14]. Forecasting results indicated that the model had high prediction efficiency. Seyyed et al. used gene expression programming to design a new model for the prediction of the compressive strength of high performance concrete (HPC) mixes [15]. Experiments showed that the prediction performance of the optimal GEP model is better than that of the regression models.

**(4) Security assessment.** In security assessment, Khattab et al. introduced gene expression programming into power system static security assessment [16]. Their algorithm showed superiority in static security assessment compared with other algorithms.

Based on these references, we know that function mining is the core of gene expression programming and that the application is very wide. With the development of data collection technology, more and more data sets are characterized by complexity, high dimensionality and massive scale. Function mining based on centralized GEP or improved algorithms leads to a significant decrease in performance. To mine a function for complex, massive and high-dimensional data sets on the basis of traditional gene expression programming, this paper presents distributed function mining for gene expression programming based on fast reduction (DFMGEP-FR), which is combined with a rough set and grid service.

This paper makes the following contributions: (1) It presents fast attribution reduction for the binary search algorithm (FAR-BSA) to quickly find the optimal reduction; (2) it solves the generation of a global function model in distributed function mining and provides consistent replacement of the local data model (CRLDM); (3) on the basis of FAR-BSA and CRLDM, it proposes forward distributed function mining for GEP on fast reduction (DFMGEP-FR); and (4) it describes simulated experiments that have been performed and provides performance analysis results.

The remainder of this paper is organized as follows. Section 2 introduces fast attribution reduction on a binary search algorithm. Section 3 addresses DFMGEP-FR. Section 4 presents experiments and performance analysis. Finally, conclusions are given in Section 5.

## Fast Attribution Reduction on a Binary Search Algorithm

### 1. Problem description

#### Example 1

Considering the following *isolet* data set in UCI standard datasets [17]. The data set contains 617 condition attributes, 26 classification decision attributes, and 6238 instances. The function model, shown in formula (1), was mined by a traditional GEP algorithm according to the parameters in Table 1. Where E, S, C, T and L represents exp, sin, cos, tan, and log, respectively, in mathematics. The flow of the traditional GEP algorithm is shown in Fig 1.

**Fig 1:** The flow chart of traditional GEP.

**Table 1:** The parameters of GEP.

Function set	+-*/ESCT
Variable set	[*x*_0_ − *x*_616_]
Link function	+
Number of genes	3
Gene head length	6
Population size	500
Mutation rate	0.044
IS transposition rate	0.3
RIS transposition rate	0.3
Gene transposition rate	0.1
One-point recombination rate	0.3
Two-point recombination rate	0.3
Gene recombination rate	0.1
Fitness function	$f_{i}=\sum_{j=1}^{n}\left(R-|P_{ij}-T_{j}|\right)$

$$10.0007+e^{e^{x_{176}}}+e^{x_{200}}+e^{x_{300}}+x_{533}+x_{200}+x_{238}+x_{260}+x_{298}+x_{300}+x_{424}+4*x_{432}+x_{590}$$ (1)

From formula (1), it is evident that for a complex, massive and high-dimensional data set, the function mined by the traditional GEP is complex, and thus, it is difficult to explain the specific meaning. At the same time, the GEP can also reduce condition attributions, but the reduction in the condition attributions by GEP has randomness and could not be explanatory.

To better mine and analyze high-dimensional data sets, attribution reduction is first performed. We know that when the sample data set is based on random sampling, redundant attributes of sample datasets are inevitable. However, these redundant attributes both increase the storage space and interfere with the user to make a correct and simple decision. In essence, attribute reduction is to reduce the redundant attributes of a sample dataset to reduce the computational complexity of the sample data processing. The existing methods for attribution reduction include principal component analysis (PCA), singular value decomposition (SVD), rough set (RS), and others; attribution reduction based on PCA and SVD inevitably result in the loss of part of the decision information, while attribution reduction based on RS does not change the decision rules of the original data set. Traditional attribution reduction algorithms based on RS do not quickly obtain the optimal reduction. Many scholars present new algorithms based on RS to decrease the time complexity for solving the optimal reduction [18,19]. Due to the diversity and equivalence of the optimal reduction, any of the optimal reductions must be solved to meet the requirements with which GEP mines complex and high-dimensional data sets. Thus, this paper presents fast attribution reduction on a binary search algorithm (FAR-BSA) to solve an optimal reduction quickly. Because FAR-BSA is based on RS, attribution reduction based on FAR-BSA does not change the decision rules of the original data set.

### 2. Preliminaries

To understand attribution reduction based on a rough set, we shall first briefly introduce the related concepts for a rough set in this paper [19].

**Definition 1.** Let the data table be *T* = < *U*,*C*∪*D*,*V*,*f* >, *C*∪*D* = *R*, where *U*, *C*, *D*, *V* = ∪*v*_*r*_, *r* ∈ *R* and *f*: *U*×*R*→*V* represent the data set, condition attribution set, decision attribution set, attribution value set and information function, respectively, and ∀*r* ∈ *R*, *x* ∈ *U*, *f*(*x*,*r*) ∈ *v*_*r*_. Data table *T* is called the decision table.

**Definition 2.** Let the decision table be *T* = < *U*,*C*∪*D*,*V*,*f* >. ∀*P* ⊆ *R*, *r* ∈ *P*, *R* = *C*∪*D*, and *x*, *y* ∈ *U* if and only if *f*(*x*,*r*) = *f*(*y*,*r*), and then, x and y are indiscernible and denoted by *IND*(*P*) = {(*x*,*y*) ∈ *U* | *r* ∈ *P*, *f*(*x*,*r*) = *f*(*y*,*r*)} or *U*/*P*.

**Definition 3.** Let the decision table be *T* = < *U*,*C*∪*D*,*V*,*f* >, *C*∪*D* = *R*. For all *X* ⊂ *U*, *R*-the lower approximations of *X* is denoted as *R*___(*X*), where *R*___(*X*) = ∪{*Y*_*i*_⊂*U* / *IND*(*R*): *Y*_*i*_⊂*X*}.

**Definition 4.** Let the decision table be *T* = < *U*,*C*∪*D*,*V*,*f* >, *C*∪*D* = *R*, For all *X*⊂*U*; then, the *R*-positive region of *X* is denoted as *POS*_*R*_(*X*), where *POS*_*R*_(*X*) = *R*___(*X*).

**Definition 5.** Let the decision table be *T* = < *U*,*C*∪*D*,*V*,*f* >. Then, the dependence degree between the condition attribution *C* and decision attribution *D* is denoted by *r*_*C*_(*D*), where $r_{C}(D)=\frac{card(POS_{C}(D))}{card(U)}$, and where *card*(*U*) represents the number of collections *U*.

**Definition 6.** Let the decision table be *T* = < *U*,*C*∪*D*,*V*,*f* >. If *r*_*C*_(*D*) = 1, then *T* is said to be consistent.

**Definition 7.** Let decision table *T* = <*U*,*C*∪*D*,*V*,*f*> be consistent. For condition attribution *c* ⊂ *C*, if *POS*_*C*_(*D*) = *POS*_*C*−{*c*}_(*D*), the condition attribution *c* is reducible.

**Property 1.** Let decision table *T* = <*U*,*C*∪*D*,*V*,*f*> be consistent. For condition attribution *c* ⊂ *C*, if *POS*_*C*_(*D*) = *POS*_*C*−{*c*}_(*D*), then *T*' = <*U*,*C*-{*c*}∪*D*,*V*,*f*>, which reduces condition attribution *c* consistently.

**Proof.** According to Definition 6, for consistent decision table *T* = < *U*,*C*∪*D*,*V*,*f* >,

$$r_{C}(D)=\frac{card(POS_{C}(D))}{card(U)}=1$$ (2)

According to the known conditions, Eq (3) holds:

$$r_{C\text{-}\{\text{c}\}}(D)=\frac{card(POS_{C\text{-}\{\text{c}\}}(D))}{card(U)}=\frac{card(POS_{C}(D))}{card(U)}$$ (3)

From (2) and (3), *r*_*C*-{*c*}_(*D*) is equal to 1, i.e., *T*' = <*U*,*C*-{*c*}∪*D*,*V*,*f*>, which reduces condition attribution *c* consistently.

**Definition 8.** Let decision table *T* = <*U*,*C*∪*D*,*V*,*f*>. *C*_1_, *C*_2_, …, *C*_*n*_ is the reduction of *T*, where *C*_1_, *C*_2_, …, *C*_*n*_ contain i, j, p condition attributions, respectively. Reduction *C*_*i*_(*i* = 1,2,…,*n*), which contains the minimum number of condition attributions, is called the optimal reduction.

**Lemma 1.** Let decision table *T* = <*U*,*C*∪*D*,*V*,*f*> be consistent, where *S* is a subset of condition attribution set *C* and is recorded as *S*⊂*C*. If S is not a reduction, then ∀*S*' ⊂ *S* is not a reduction either.

**Proof.** Suppose that ∀*S*' ⊂ *S* ⊂ *C* is a reduction; then, from Property 1, we know that decision table *T* is still consistent after *S*' is removed from *C*. In addition, because *S*' ⊂ *S*, then (*C* − *S*) ⊂ (*C* − *S*'). According to Definition 7 and the known conditions, decision table *T* must be consistent after *S*' is removed from *C*. Then, from Property 1, we know that for *S* ⊂ *C*, *S* is said to be reducible, also. This conclusion is inconsistent with the known conditions. Thus, the original proposition is correct.

### 3. Algorithm Description

To better mine the function model for high-dimensional sample data sets by GEP, the reduction of high-dimensional data sets must be performed to rapidly solve the optimal reduction. Thus, this paper presents fast attribution reduction on a binary search algorithm (FAR-BSA).

#### Example 2

Let the decision table be *T* = <*U*,*C*∪*D*,*V*,*f*>, where *C* = {*x*_1_, *x*_2_, *x*_3_, *x*_4_}, and the process of solving the optimal reduction based on binary search is as follows.

1. First, let *m* equal 2, looping through all of the reductions to include two condition attributions in *C*.
2. Suppose that when *m* equals 2, reduction exists. Then, the number of condition attributions in the optimal reduction is between 1 and 2. Let *m* equal 1 again, looping through all reductions to include one condition attribution in *C*. If reduction exists when *m* equals 1, then the reduction is an optimal reduction and includes one condition attribution or two condition attributions.
3. Suppose that when *m* equals 2, reduction does not exist. Then, the number of condition attributions in the optimal reduction is between 3 and 4. Let *m* equal 3 again, looping through all of the reductions to include three condition attributions in *C*. If reduction exists when *m* equals 3, then the reduction is an optimal reduction and includes three condition attributions, or the condition attribution collection *C* is itself the optimal reduction. According to the above description, the basic steps of FAR-BSA are shown as follows:

Algorithm 1: FAR-BSA (T).

Input: *T* = <*U*,*C*∪*D*,*V*,*f*>, where condition attribution collection *C* = {*x*_1_,*x*_2_,…,*x*_*n*_};

Output: bestReduction;

1. int *m* = ⌊*n*/2⌋;

2. if (*C*_*m*_ is reduction) {

3.    if (*m* = 1) {bestReduction = *C*_*m*_; return bestReduction; break;}

4.    else if (*m* = *n*) {bestReduction = *C* = *C*_*n*_; return bestReduction; break;}

5.    else {*m* = ⌊*m*/2⌋; goto 2;}}

6. else {

7.    *m* = ⌊(*m* + *n*)/2⌋; goto 2;}

8. return bestReduction;

where *C*_*m*_ contains *m* condition attributions. Note that in this paper, we assume that the sample decision table is coordinated. In FAR-BSA, the time complexity of computing the condition attribution combination is $O(\log_{2}^{m})(1\leq m\leq n)$ maximally. According to the coordination of the sample decision table, the time complexity of computing a reduction is *O*(|*U*|). Thus, the time complexity of solving the optimal reduction is $O(|U|\times \log_{2}^{m})$.

## Distributed Function Mining for Gene Expression Programming on Fast Reduction

### 1. Algorithm idea

On the basis of FAR-BSA, the dimension of the data set could be effectively reduced. Owing to the characteristics of the rough set itself, dimension reduction does not change the inherent property of the original data set. At the same time, for massive or distributed data sets, centralized mining will lead to a series of problems such as security, privacy and mining efficiency and requires a large amount of network bandwidth.

Grid is a high performance and distributed computing platform with good self-adaptability and scalability and provides favorable computing and analysis capability for massive and distributed data sets. Grid could provide strong analysis and computing power with distributed data mining and knowledge discovery. In view of the advantages of grid computing, on the basis of FAR-BSA, this paper presents distributed function mining for gene expression programming based on fast reduction (DFMGEP-FR), which is combined with a rough set and grid service.

Suppose that data on each grid node is homogeneous in this paper. The algorithm idea is divided into sub-processes. First, the FAR-BSA and GEP algorithm are wrapped as grid services and deployed on each grid node. At the same time, the attributions of distributed data sets are reduced on the different grid nodes, and distributed function mining for data sets after reduction is performed in parallel by calling the GEP grid service. Finally, the local function model from each grid node is integrated into the global function model.

### 2. Function consistency replacement algorithm

For generating a global data model from the local data model, consistency replacement of the local data model (CRLDM) is proposed. To more clearly describe the idea of CRLDM, definition 9 is given as follows.

**Definition 9.** Suppose that there are *N* grid nodes and *K*_*i*_,*i*∈[1,*N*] (abbreviated *K*_*i*_) sample data in the *i-*th grid node; each sample data includes *n* condition attributions *x*_*i*_,*i*∈[1,*n*] and a decision attribution *y*_*j*_, *j* ∈ [1,*K*_*i*_]. In addition, *f*_*i*_(*x*_1_,*x*_2_,……,*x*_*n*_),*i*∈[1,*N*] mined on the *i-*th grid node is abbreviated as *f*_*i*_. For each row of sample data in the *i-*th grid node, if |*y*_*j*_ − *f*_*i*_| < *δ*, then the *j-*th sample data on the *i*th grid node *δ*-fit *f*_*i*_.

From Definition 9, we know that there were *S*_*i*_,*i* ∈ [1,*N*] (abbreviated *S*_*i*_) sample data that *δ*-fitted function *f*_*i*_ when *f*_*i*_ fitted the *K*_*j*_ sample data. Based on the same principle, when *f*_*j*_ fitted the *K*_*i*_ sample data, there were *S*_*j*_ sample data that *δ*-fitted function *f*_*j*_, where *i* ≠ *j*. The following properties then appear:

**Property 2.** (1) When *K*_*i*_ = *S*_*j*_ or *K*_*j*_ = *S*_*i*_, *f*_*i*_ completely fit *K*_*j*_ or *f*_*j*_ completely fit *K*_*i*_; in other words, *f*_*i*_ and *f*_*j*_ are equivalent. (2) When *K*_*i*_ = *K*_*j*_, if *S*_*j*_ < *S*_*i*_, then *f*_*i*_ replaces *f*_*j*_; otherwise, *f*_*j*_ replaces *f*_*i*_. (3) When *K*_*i*_ > *K*_*j*_, if $(\frac{S_{j}}{K_{i}}-\frac{S_{i}}{Kj})<0$, then *f*_*i*_ replaces *f*_*j*_; otherwise, *f*_*j*_ replaces *f*_*i*_. (4) When *K*_*i*_ < *K*_*j*_, if $(\frac{S_{i}}{Kj}-\frac{S_{j}}{K_{i}})<0$, then *f*_*j*_ replaces *f*_*i*_; otherwise, *f*_*i*_ replaces *f*_*j*_.

**Proof**. (1) Property 2-(1) is clearly established. (2) When *K*_*i*_ = *K*_*j*_, if *S*_*j*_ < *S*_*i*_, then for the same amount of sample data, the number of sample data instances that *f*_*i*_ fits is more than *f*_*j*_. Thus, *f*_*i*_ replaces *f*_*j*_, and vice versa. (3) When *K*_*i*_ > *K*_*j*_, if $(\frac{S_{j}}{K_{i}}-\frac{S_{i}}{Kj})<0$, then the number of sample data instances that *f*_*i*_ fits is more than *f*_*j*_. Thus, *f*_*i*_ replaces *f*_*j*_, and vice versa. (4) The process for the proof is the same as (3).

The consistency replacement algorithm of the local data model is shown as follows:

Algorithm 2: Consistency Replacement of the Local Data Model (CRLDM)

Input: *f*_*i*_(*x*_1_,*x*_2_,…,*x*_*m*_),*i*∈[1,*N*];

Output: Global function expression;

Algorithm CRLDM (*f*_*i*_(*x*_1_,*x*_2_,……,*x*_*m*_))

Begin {

1. For any *i* ≠ *j*,*i*,*j* ∈ [1,*N*], the number of sample data instances for which *f*_*i*_ fits *K*_*j*_ and *f*_*j*_ fits *K*_*i*_ is calculated.

2. if (*K*_*i*_ = *S*_*j*_ or *K*_*j*_ = *S*_*i*_) {*f*_*i*_ replaces *f*_*j*_ or *f*_*j*_ replaces *f*_*i*_;}

3. if (*K*_*i*_ = *K*_*j*_){

4.    if (*S*_*j*_ < *S*_*i*_) {*f*_*i*_ replaces *f*_*j*_;} else {*f*_*j*_ replaces *f*_*i*_}}

5. else if (*K*_*i*_ > *K*_*j*_) {

6.    if ($(\frac{S_{j}}{K_{i}}-\frac{S_{i}}{Kj})<0$) {*f*_*i*_ replaces *f*_*j*_;} else {*f*_*j*_ replaces *f*_*i*_;}}

7.    else {

8.    if ($(\frac{S_{i}}{Kj}-\frac{S_{j}}{K_{i}})<0$) {*f*_*j*_ replaces *f*_*i*_;} else {*f*_*i*_ replaces *f*_*j*_;}}

End

To better evaluate the performance of the global function, a definition for the global fitting error is given in this paper.

**Definition 10.** For *N* grid nodes, let the global function expression be *f*(*X*), where there are *K*_*i*_,*i* ∈ [1,*N*] sample data in the *i*th node. If the *E*_*i*_ sample data are not fitted when *f*(*X*) fits *K*_*i*_, then $GFE=\frac{\sum_{i=1}^{N}E_{i}}{\sum_{i=1}^{N}K_{i}}\times 100\%$ is called the global fitting error (GFE).

The aim of the function consistency replacement algorithm for the local data model is to attempt to keep the global fitting error unchanged; thus, the global function expression by distributed function mining fits the sample data for centralized mining as much as possible.

### 3. Description of DFMGEP-FR

A whole algorithm that is based on grid service includes the client and server. DFMGEP-FR is described from the perspective of the client and server. The description of the whole algorithm is as follows:

Algorithm 3: Distributed Function Mining for GEP on Fast Reduction (DFMGEP-FR)

Input: Sample data decision table *T* = <*U*,*C*∪*D*,*V*,*f*>, Grid service address of GEP (GEPGSH), GEP parameters (GEPParas);

Output: Global function expression (GlobalFunction);

Begin {

Server:

1. ReceivePara(T, GEPParas,i,GEPGSH);// Sample data, GEPParas, grid node *i*, GEPGSH are received from client.

2. FAR-BSA (T);//FAR-BSA is called to reduce the condition attribution of the sample data, and the sample data are returned after reduction.

3. Initialization of Population S;//Initializing population of GEP according to the sample data after reduction.

4. LocalFunction(i) = GEP(S);//GEP algorithm is applied to the sample data after reduction, and the local function expression is returned.

Client:

5. T = Read(SampleData);//Reading sample data and constructing Sample data decision table *T*.

6. int gridcodes = SelectGridCodes();//Selecting grid node of deploying GEP algorithm service.

7. for (int i = 0; i<gridcodes; i++) {

8.    TransPara(T,GEPParas,i,GEPGSH);//Transmitting the parameters to the server.

9.    TransService (LocalFunction[i]);}//Returning the local function expression of the *i*th grid node to the client.

10. CRLDM(LocalFunction);//Calling the consistency replacement algorithm of the local data model to obtain the global function expression.

11. return GlobalFunction;}

End

From Algorithm 3, we know that the execution time of the DFMGEP-FR algorithm includes the time for the attribute reduction, the time for function mining based on the GEP of each grid node and the time for transmission parameters and replacement of local function expression. In a LAN environment, the time for the transmission parameters can be ignored, and the integration of the local function expression does not affect the performance of the distributed function mining. At the same time, due to the use of fast attribution reduction based on a binary search algorithm, the dimension of the sample data sets on each grid node is greatly reduced to further reduce the time complexity of the function mining based on GEP.

Let the total time of the DFMGEP-FR algorithm be *t*_*total*_, the time for the reduction of the sample data set be *t*_*reduction*_, the time for the function mining on each grid node be *t*_*FMGEP*_, the time of the data transmission be *t*_*transParas*_, and the time of the local model replacement be *t*_*CRLDM*_. Then, Eq (4) is as follows:

$$t_{total}=t_{reduction}+t_{FMGEP}+t_{transParas}+t_{CRLDM}$$ (4)

The time required for DFMGEP-FR can be very convenient for the calculation and evaluation of Eq (4).

## Experimental Results and Discussion

To verify the effectiveness of the DFMGEP-FR, this paper performs simulation experiments in a LAN environment on a cluster of 2* hexa-core 2.01G Xeon CPUs. Two simulation experiments were performed on the following platform: WS-Core+Eclipse+Tomcat+Ant+Redhat Linux 9.

All of the data sets in this paper are also available on the UCL machine learning archive [17]. Currently, there are 311 data sets in the entire UCI set. There are 97 data sets for which the number of attributions is greater than 20 and the number of instances is greater than 1500. Due to the limitations of the experimental environment, it is not possible to perform experiments on 97 data sets. Thus, according to the requirements of the algorithm for the number of attributions and scale, this paper chooses six data sets from the 97 data sets. The six data sets that we used are shown in Table 2. In addition, they were selected to have various numbers of condition attributions (from 16 to 617), decision attributions (from 1 to 26), and instances (from 5000 to 67557), and they are used as representative samples of the problems that FAR-BSA can address.

**Table 2:** Data sets used in our experiments.

Data Set	Number of condition attributions	Number of decision attributions	Number of instances
bank	16	1	45211
waveform	21	3	5000
mushroom	22	2	8124
connect-4	42	3	67557
musk	168	2	6598
isolet	617	26	6238

### Experiment 1

To illustrate the effect of attribution reduction for high-dimensional function mining, this paper uses centralized GEP to mine function models for six data sets before and after reduction in Table 2. The number of optimal reductions based on FAR-BSA, the attribute reduction algorithm based on the positive region (AR-PR), the attribute reduction algorithm based on a discernable matrix (AR-DM), mRMR [20], PCA and SVD are shown in Fig 2. A comparison of the average time-consumption and the standard deviation of the time-consumption between FAR-BSA and other reduction algorithms is shown in Table 3. Table 4 shows a comparison of the average time-consumption and the standard deviation of the time-consumption by the centralized function mining for six data sets before and after reduction under the condition that the centralized GEP algorithm runs 10 times.

**Fig 2:** Comparison of the number of optimal reductions under different attribution reduction algorithms.

**Table 3:** Comparison of the average time-consumption and standard deviation of the time-consumption between FAR-BSA and other reduction algorithms.

	**Average time-consumption of attribution reduction (S)**					
	FAR-BSA	AR-PR	AR-DM	PCA	SVD	mRMR
bank	722	2865	924	120	124	2868
waveform	401	891	524	151	151	889
mushroom	422	911	698	169	166	920
connect-4	831	3611	1821	870	887	3598
musk	496	3247	1040	11354	12659	3244
isolet	560	3918	2005	25032	26352	3901
	**Standard deviation of the time-consumption**					
	FAR-BSA	AR-PR	AR-DM	PCA	SVD	mRMR
bank	0.147	0.17	0.161	0.1741	0.1841	0.14
waveform	0.254	0.2701	0.2601	0.2587	0.2687	0.2487
mushroom	0.201	0.23	0.2231	0.2209	0.2309	0.2027
connect-4	0.276	0.301	0.2913	0.3111	0.3121	0.2801
musk	0.317	0.356	0.34	0.3345	0.356	0.3099
isolet	0.447	0.553	0.531	0.5409	0.55	0.4499

**Table 4:** Comparison of the average time-consumption and standard deviation of the time-consumption by centralized function mining for six data sets before and after reduction.

	**Average time-consumption of centralized function mining by GEP (S)**						
	before reduction	after reduction based on the following algorithms					
		FAR-BSA	AR-PR	AR-DM	PCA	SVD	mRMR
bank	2735	822	896	895	871	865	870
waveform	1925	501	511	512	505	503	502
mushroom	2439	522	539	561	535	534	533
connect-4	4165	931	2012	3099	998	992	1001
musk	3619	616	813	1012	762	756	761
isolet	4918	730	941	1112	901	900	876
	**Standard deviation of the time-consumption**						
	before reduction	after reduction based on the following algorithms					
		FAR-BSA	AR-PR	AR-DM	PCA	SVD	mRMR
bank	0.11	0.1337	0.1541	0.1641	0.1655	0.161	0.1378
waveform	0.23	0.241	0.2487	0.2687	0.2801	0.2601	0.2487
mushroom	0.2	0.211	0.2209	0.2259	0.2401	0.2231	0.2127
connect-4	0.269	0.2811	0.3311	0.3321	0.301	0.2913	0.2859
musk	0.3619	0.321	0.3345	0.356	0.356	0.34	0.316
isolet	0.4918	0.447	0.5409	0.55	0.6353	0.531	0.4499

From Fig 2, for all of the datasets, the number of optimal reductions based on FAR-BSA, AR-PR, AR-DM and mRMR is less than the number of optimal reductions based on PCA and SVD. For the bank, waveform, mushroom, and connect-4 datasets, compared with AR-PR, AR-DM and mRMR, the number of optimal reductions based on FAR-BSA does not change. These findings demonstrate that attribution reduction based on a rough set is effective. For musk, the number of optimal reductions based on FAR-BSA decreases, respectively, by 15.38% and 26.67%, compared to PCA and SVD, while that for isolet decreases by 8.7% and 12.5% compared to PCA and SVD (respectively). However, compared with mRMR, the number of optimal reductions based on FAR-BSA increases by 9.09% and 9.52% (respectively). In Table 3, it is shown that FAR-BSA outperforms AR-PR, AR-DM and mRMR for all of the data sets, and the average time-consumption based on FAR-BSA decreases by 74.83%, 54.99%, 54.13%, 76.99%, 84.72% and 85.71% maximally for the bank, waveform, mushroom, connect-4, musk and isolet datasets, respectively. However, for the bank, waveform, and mushroom datasets, PCA and SVD are better than FAR-BSA. This is mainly because the maximum time complexity of FAR-BSA is $O(|U|\times \log_{2}^{m})(1\leq m\leq \left|C\right|)$, while the time complexity of AR-PR, AR-DM, mRMR, PCA and SVD is *O*(|*C*|×|*U*|), $O(|C|\times \frac{\left|U\right|}{2})$, *O*(|*C*|×|*U*|), *O*(|*C*|^3^), *O*(|*C*|^3^), respectively. From Table 3, it is shown that for the bank, waveform, mushroom, connect-4, musk and isolet datasets, the maximum standard deviation of the time-consumption based on FAR-BSA, AR-PR, AR-DM, PCA, SVD and mRMR is 0.1841, 0.2701, 0.2309, 0.3121, 0.356 and 0.55, respectively. This finding means that the time-consumption of the six attribution reduction algorithms is relatively stable and close to the average value of the time-consumption under the condition that these algorithms run 10 times. Table 4 shows that before and after the attribution reduction, the average time-consumption based on centralized GEP for the bank, waveform, mushroom, connect-4, musk and isolet datasets decreases maximally by 69.95%, 73.97%, 78.6%, 77.65%, 82.98% and 85.16%, respectively. From Table 4, we can see that the maximum standard deviation of the average time-consumption based on centralized GEP for the bank, waveform, mushroom, connect-4, musk and isolet datasets before and after reduction is 0.1655, 0.2801, 0.2259, 0.3321, 0.3619 and 0.6353, respectively. The research means that the time-consumption of the function mining based on centralized GEP for the bank, waveform, mushroom, connect-4, musk and isolet datasets is relatively stable and close to the average value for the time-consumption under the condition that these algorithms were run 10 times.

### Experiment 2

From experiment 1, it is obvious that for massive and complicated data sets, centralized function mining based on GEP is still a very difficult task. To solve this problem, experiment 2 uses a grid platform to design a parallel and distributed function mining algorithm. In experiment 2, the waveform, mushroom, connect-4, and musk datasets are selected from Table 2. The four data sets reflect not only the complexity of the data set but also the scale of the data set. The parameters of the algorithm are shown in Table 5. A comparison of the average time-consumption and standard deviation of the time-consumption among DFMGEP-FR, parallel GEPSA [21] and centralized GEP is shown in Table 6. In these cases, DFMGEP-FR and parallel GEPSA were run under the environment of ten grid nodes, and all of the algorithms were run 10 times. The fitting degree between the real value and model value of the waveform, mushroom, connect-4, and musk dataset is shown in Fig 3. Fig 4 shows a comparison of the global fitting error for the waveform, mushroom, connect-4, and musk datasets for 1 to 10 grid nodes.

**Fig 3:** Comparison between the model value and real value for four test data sets for DFMGEP-FR, parallel GEPSA and centralized GEP.

**Fig 4:** Comparison of the global fitting error for all of the tested datasets under different grid nodes.

**Table 5:** Parameters of DFMGEP-FR.

function set	+-*/SCLE
variable set	[*x*_0_ − *x*_4_] (for waveform)
	[*x*_0_ − *x*_4_] (for mushroom)
	[*x*_0_ – *x*_2_] (for connect-4)
	[*x*_0_ – *x*_10_] (for musk)
link function	+
number of genes	3
gene head length	9
population size	100
mutation rate	0.044
IS transposition rate	0.3
RIS transposition rate	0.3
gene transposition rate	0.1
one-point recombination rate	0.3
two-point recombination rate	0.3
gene recombination rate	0.1
fitness function	$f_{i}=\sum_{j=1}^{n}\left(100-|P_{ij}-T_{j}|\right)$
the number of generations	50000
the number of grid nodes	10

**Table 6:** Comparison of the average time-consumption and standard deviation of the time-consumption between DFMGEP-FR and other algorithms.

	**Average time-consumption of three algorithms(S)**		
	DFMGEP-FR	Centralized GEP	Parallel GEPSA
waveform	210	1925	240
mushroom	272	2439	297
connect-4	592	4165	655
musk	251	3619	291
	**Standard deviation of the time-consumption**		
	DFMGEP-FR	Centralized GEP	Parallel GEPSA
waveform	0.011	0.014	0.023
mushroom	0.013	0.019	0.0211
connect-4	0.17	0.18	0.168
musk	0.208	0.2	0.201

Table 6 shows that on the basis of mining the ideal function, for the waveform, mushroom, connect-4 and musk datasets, DFMGEP-FR outperforms all of the other algorithms in terms of the average time-consumption. For the waveform, mushroom, connect-4 and musk datasets, compared with centralized GEP, the average time-consumption based on DFMGEP-FR drops by 89.09%%, 88.85%, 85.79% and 93.06%, respectively. However, for the waveform, mushroom, connect-4 and musk datasets, compared with parallel GEPSA [21], the average time-consumption based on DFMGEP-FR decreases by 12.5%, 8.42%, 9.62% and 13.75%, respectively. This is mainly because for the waveform, mushroom, connect-4 and musk datasets, DFMGEP-FR performs the attribution reduction in advance, to greatly decrease the dimension of the sample data sets. At the same time, in the grid environment, the number of data sets is reduced on each grid node. In the LAN, network transmission delay among grid nodes is basically negligible, and thus, the time that is consumed by function mining based on DFMGEP-FR is greatly decreased. At the same time, Table 6 shows that the maximum standard deviation of the average time-consumption based on DFMGEP-FR, parallel GEPSA [21] and centralized GEP for the waveform, mushroom, connect-4 and musk datasets is 0.23, 0.211, 0.18 and 0.2080, respectively. It is shown that ten time-consumption values for the function mining based on DFMGEP-FR, parallel GEPSA [21] and centralized GEP for the waveform, mushroom, connect-4 and musk datasets yield approximately the average value. From the perspective of the effects of function mining, function expression by DFMGEP-FR is simpler than by centralized GEP and parallel GEPSA [21]. For the waveform, mushroom, connect-4 and musk datasets, the function expression based on DFMGEP-FR is shown in formulas (5), (6), (7) and (8), respectively.

$$0.2128+\frac{0.9015}{6.1804+x_{0}-x_{2}+x_{3}-x_{4}}+\sin(\sin(\frac{0.7041}{6.1804+x_{1}}))$$ (5)

$$2x_{3}-x_{2}(x_{4}-x_{0})+x_{1}(x_{1}-x_{2})+e^{x_{1}}(x_{1}-x_{4})$$ (6)

$$0.02798x_{0}{}^{2}x_{1}x_{2}+2\cos(x_{0}{}^{2}x_{2}{}^{3})$$ (7)

$$10.0007x_{9}x_{1}x_{5}(x_{10}x_{2}x_{6}+x_{0}x_{3}x_{8}+x_{4}x_{7}x_{8})$$ (8)

From Fig 3, by using DFMGEP-FR, we can see that the maximum error between the model value and real value of the waveform, mushroom, connect-4 and musk sets is 1.5463, 2, 2 and 0.0263, and the minimum error is 0.1404, 0, 0 and 0, respectively; by using parallel GEPSA, the maximum error between the model value and real value for the waveform, mushroom, connect-4 and musk datasets is 1.5789, 3.61, 2.21 and 0.02971, respectively, and the minimum error is 0.4496, 0, 0 and 0, respectively; by using centralized GEP, the maximum error between the model value and real value for the waveform, mushroom, connect-4 and musk datasets is 1.664, 3.15, 2.43 and 0.03171, respectively, and the minimum error is 0.3227, 0, 0 and 0, respectively. It can be observed that the model that is based on DFMGEP-FR has good prediction accuracy in contrast to parallel GEPSA and centralized GEP. From Fig 4, we know that when the number of grid nodes increases from 1 to 3, the global fitting error apparently decreases. For the waveform, mushroom, connect-4 and musk datasets, the global fitting error of DFMGEP-FR drops by 3.34%, 3.31%, 6.73% and 5.87%, respectively. With an increase in the number of grid nodes, the global fitting error remains unchanged. When the number of grid nodes increases to 9, for the waveform, mushroom, connect-4 and musk datasets, the global fitting error of DFMGEP-FR increases by 5.26%, 0.97%, 1.64% and 1.49%, respectively. This is because for data sets of a specific size, the greater the number of grid nodes that are involved in the function mining, the more easily the global function model is obtained. However, with an increase in the number of grid nodes, a low number of data samples on each node make the local function model more dispersed, in such a way that it is difficult for the global function model to fit most of the sample data. In addition, the increasing grid nodes also improve the time consumption that is required in integrating the local function model and the whole algorithm.

## Conclusions

To better solve the defects in massive and high-dimensional function mining, this paper proposes fast attribution reduction on a binary search algorithm (FAR-BSA). This algorithm applies the idea of a binary search to attribution reduction, to greatly decrease the time complexity of solving the optimal attribution reduction. On the basis of FAR-BSA, distributed function mining for GEP on fast reduction (DFMGEP-FR) is present. Simulated experiments show that for massive and high-dimensional data sets, FAR-BSA outperforms all of the other algorithms. Moreover, the time consumption of DFMGEP-FR is less than parallel GEPSA and traditional GEP. With an increase in the number of grid nodes, the global fitting error of DFMGEP-FR first decreases and then increases gradually.

DFMGEP-FR makes full use of distributed computing resources to improve the computing efficiency. In DFMGEP-FR, fast attribution reduction on a binary search algorithm is still performed on a single PC server. However, with increasing condition attributions of data sets, the average time consumption of the centralized attribution reduction algorithm will increase continuously. Thus, the distributed attribution reduction algorithm will become an important direction of study in the future.
